The article "4-Methoxydalbergione Elicits Anticancer Effects by Upregulation of GADD45G in Human Liver Cancer Cells" was published in 2023. Journal: J Healthc Eng.

# 4-Methoxydalbergione Elicits Anticancer Effects by Upregulation of GADD45G in Human Liver Cancer Cells

**DOI:** 10.1155/2023/6710880

**Published:** 2023-02-01

**Authors:** Liping Zeng, Yuqi Qin, Xiaomin Lu, Xianlei Fang, Jianghua Huang, Cong Yu, Zhen-Bo Feng

**Affiliations:** ^1^Department of Pathology, The First Affiliated Hospital of Guangxi Medical University, Nanning 530021, Guangxi Zhuang Autonomous Region, China; ^2^Department of Pathology, Jiangbin Hospital of Guangxi Zhuang Autonomous Region, Nanning 530021, Guangxi Zhuang Autonomous Region, China; ^3^Department of Pathology, Hunan University of Medicine, Huaihua 418000, Hunan, China

## Abstract

**Background:**

4-Methoxydalbergione (4MOD) is a flavonoid isolated from the heartwood of Dalbergia. Studies have demonstrated that 4MOD exerts anticancer activities on bladder cancer and astrocytoma. However, the anticancer activity of 4MOD in hepatocellular carcinoma (HCC) remains unknown. This study aims to examine its anticancer activities and mechanisms in human liver cancer cells.

**Methods:**

CCK-8, colony forming, wound healing, transwell migration, and AnnexinV/PI assays were used to assess the anticancer effects of 4MOD in HCC cells. RNA sequencing (RNA-Seq) was selected to explore the possible mechanisms underlying the anti-HCC activity of 4MOD. The mRNA expression levels of target genes were verified through quantitative real-time PCR (qRT-PCR). A lentiviral shRNA interference technique was used to silence GADD45G expression. GADD45G knockdown was employed to confirm the crucial role of GADD45G in the 4MOD-mediatedanti-HCC effects.

**Results:**

4MOD inhibited HCC cells' proliferation and migration and promoted tumor cell apoptosis. RNA-Seq and qRT-PCR analyses revealed that 4MOD treatment increased GADD45G expression. Silencing GADD45G reversed 4MOD-mediated inhibition of proliferation, migration, and promotion of apoptosis.

**Conclusions:**

Our findings show that 4MOD elicits anti-HCC effects by upregulating GADD45G expression and could be a valuable anticancer agent for liver cancer.

## 1. Introduction

As the predominant histological type of primary liver cancer, hepatocellular carcinoma (HCC) seriously endangers people's health. According to global cancer statistics 2020, there are about 906,000 new cases of HCC and 830,000 deaths worldwide every year [1]. Currently, despite progress in therapeutic approaches for liver cancer such as surgery, targeted therapy, and liver transplantation, the 5-year overall survival (OS) of advanced-stage HCC patients remains only 10% [2]. Resistance to chemotherapy remains a major cause of treatment failure in advanced-stage HCC [3]. Therefore, the development of more effective antiliver cancer drugs is of clinical significance.

Currently, many natural herbal products have been proven to exhibit anticancer effects and have received considerable attention [4–7]. Flavonoids, a complex class of bioactive compounds, are widely distributed in various plants, foods, and vegetables. Increasing evidence has demonstrated that flavonoids exhibit significant anti-inflammatory [8], anticancer [9], and antioxidant [10] activities. 4-Methoxydalbergione (4MOD) is a kind of flavonoid isolated from the heartwood of *Dalbergia*, with anti-inflammatory activities [11]. In addition, recent studies have revealed that 4MOD has anticancer effects on bladder cancer and astrocytoma [12, 13]. However, the anticancer activity of 4MOD in HCC remains unknown.

Growth arrest and DNA damage are inducible. The 45G (GADD45G), a member of the GADD45 family, participates in DNA damage response and cell growth arrest. Studies have confirmed that GADD45G is lowly expressed in esophageal squamous cell carcinoma, breast cancer, and acute myeloid leukemia [14–16]. It has also been reported that the upregulation of GADD45G expression induces the senescence of HCC cells [17]. Hence, GADD45G might be a novel target for HCC treatment.

Herein, we have characterized 4-Methoxydalbergione's anticancer effects on HCC cells' proliferation, migration, and apoptosis. In addition, the molecular mechanism of 4MOD's action against liver cancer was elucidated. We determined that 4MOD significantly inhibited human liver cancer cells' proliferation and migration, as well as promoting cell apoptosis through upregulation of GADD45G *in vitro*.

## 2. Materials and Methods

### 2.1. Cell Culture and Drug

Human liver cancer cells (SK-HEP-1 and HuH-7) were purchased from the National Collection of Authenticated Cell Cultures (Shanghai, China) and cultured in Dulbecco's Modified Eagle Medium (DMEM, Gibco, CA, USA) with 10% fetal bovine serum (FBS, Gibco, CA, USA) and 1% penicillin-streptomycin solution (Beyotime, Shanghai, China). 4MOD (98% purity, MW = 254.3) was obtained from Shanghai Yuanye Biotechnology Co., Ltd. (Shanghai, China). Dimethyl sulfoxide (DMSO, BioFoxx, Guangzhou, China) was used to dissolve 4MOD at an initial concentration of 50 mM.

### 2.2. CCK-8 Assay

Two thousand cells/well were planted overnight in 96-well plates (Corning, NY, USA). After incubation with different doses of 4MOD for 24, 48, or 72 hours, cell viability was measured with Cell Counting Kit 8 (CCK-8) solution (Dojindo, Kumamoto, Japan). In addition, the morphological changes of cells exposed to different doses of 4MOD for 48 h were observed and photographed.

### 2.3. Colony Forming Assay

1 × 10^3^ cells/well were planted overnight in 6-well plates (Corning, NY, USA). After treatment with or without 4MOD for 48 h, cells were incubated in a 5% CO_2_ humidified incubator for 2–3 weeks. When the colonies appeared, cells were fixed with 4% paraformaldehyde (Beyotime, Shanghai, China) and stained with crystal violet staining (Beyotime, Shanghai, China). An inverted microscope was used to count colonies.

### 2.4. Wound Healing Assay

HCC cells were grown overnight in 6-well plates to 90% confluency. We scratched the cells with a 100 *μ*L sterile pipette tip and further treated them with different concentrations of 4MOD. The different drug concentrations were diluted in DMEM containing 1% FBS. Pictures were obtained at 0, 24, and 48 h after creating the scratch wound using an inverted microscope. The area of scratches was measured using ImageJ software (MD, USA).

### 2.5. Transwell Migration Assay

After 48 h of culture with or without 4MOD, 3 × 10^4^ cells/100 *μ*L were planted into the transwell upper chamber (Corning, NY, USA) with serum-free DMEM, and the lower chamber contained 20% FBS. After 24 h of incubation, cells were fixed with 4% paraformaldehyde and stained with crystal violet staining solution. The cells at the bottom of the upper chamber were photographed at random. The numbers of cells were analyzed by ImageJ software (MD, USA).

### 2.6. Flow Cytometry Assay for Apoptosis Analysis

Cells were grown overnight in 6-well plates to 50% confluency. After 48 h of culture with or without 4MOD, cells were harvested and stained with Annexin V/PI (KeyGEN BioTECH, Jiangsu, China) in accordance with the protocol of manufacture. The cell apoptosis rate was detected by flow cytometry (Beckman Coulter, Miami, FL, USA). The FlowJo 10 software (Tree Star, Inc. Ashland, OR) was used for data analysis.

### 2.7. RNA Extraction and RNA Sequencing (RNA-Seq)

SK-HEP-1 cells (1 × 10^6^ cells/plate) were planted in 10 cm^2^ plates (Corning, NY, USA) overnight and then treated with 0 *μ*M or 20 *μ*M of 4MOD for 24 h. The total RNA was isolated from SK-HEP-1 cells using TRIzol reagent kit (Invitrogen, Carlsbad, CA, USA). The RNA-Seq was completed by Gene Denovo Biotechnology Co. (Guangzhou, China) through Illumina Novaseq6000 platform. For the differentially expressed genes' (DEGs) identification, a false discovery rate (FDR) <0.05 and an absolute log2 fold change of >1 were set as cutoff criteria. For the gene ontology (GO) enrichment analysis, Kyoto encyclopedia of genes and genomes (KEGG) pathway enrichment analysis, and gene set enrichment analysis (GSEA), FDR ≤0.05 was set as the threshold.

### 2.8. Transcriptome Validation by qRT-PCR

After treatment with or without 4MOD for 24 hours, the total RNA was isolated from HCC cells using the TRIzol reagent kit. HiScript IIIRT SuperMix for qPCR (Vazyme, Nanjing, China) was used to obtain cDNA. The cDNA products were amplified using 2X Universal SYBR Green FAST qPCR Mix (ABclonal, Wuhan, China). Primer sequences used for quantitative real-time PCR (qRT-PCR) are exhibited in Table 1. Relative mRNA expression levels of target genes were analyzed by 2^−ΔΔCt^ method. GAPDH was used as the internal reference.

### 2.9. Lentivirus Transfection

In our study, the lentiviral shRNA interference technique was used to generate human GADD45G knockdown cell lines. Lentivirus shRNA vectors were packaged and constructed by Genechem Co. Ltd (Shanghai, China). The shRNA sequences of GADD45G were 5′-GCACTGCATCCTCATTTCGAA-3′ (shGADD45G). The shRNA sequences of negative control were 5′-TTCTCCGAACGTGTCACGT-3′ (shNC).

### 2.10. Statistical Analysis

All experiments were repeated three times. Data were presented as mean ± standard deviation (SD) and analyzed by SPSS26.0 and GraphPad Prism 8.0 softwares. The student *t*-test was used for statistical comparison between two groups. A one-way ANOVA was used for statistical comparison among multiple groups. *p* values < 0.05 were considered statistically significant.

## 3. Results

### 3.1. 4MOD Inhibits the Proliferation of HCC Cells

To understand the cytotoxicity of 4MOD on HCC cells, morphological changes of cells exposed to different doses of 4MOD for 48 h were observed and photographed. We found that 4MOD could remarkably damage HCC cells. It was evident that 4MOD reduced cell numbers, destroyed cell structure, and made the cell round (Figures 1(a) and 1(b)). Furthermore, we used the CCK-8 assay to verify the cytotoxicity of 10, 20, 30, 40, and 50 *μ*M of 4MOD for 24, 48, and 72 h on HCC cells. The CCK-8 results indicated that 4MOD significantly repressed cell growth in both SK-HEP-1 and HuH-7 cells (Figures 1(c) and 1(d)). The IC_50_ values of SK-HEP-1 cells treated with 4MOD for 24, 48, and 72 h were 42.09 *μ*M, 29.33 *μ*M, and 13.38 *μ*M, respectively. The IC_50_ values of HuH-7 cells treated with 4MOD for 24, 48, 72 h were 31.16 *μ*M, 22.83 *μ*M, and 13.95 *μ*M, respectively. Interestingly, HuH-7 cells were more sensitive to 4MOD than SK-HEP-1 cells (Table 2). In the following cell function experiments, we selected 5 *μ*M, 10 *μ*M, and 20 *μ*M of 4MOD for treating SK-HEP-1 cells and 2.5 *μ*M, 5 *μ*M, and 10 *μ*M for HuH-7 cells treatment. In addition, we further evaluated the inhibitory effect of 4MOD on HCC cells by a colony-forming assay. As expected, the results revealed that the proliferation of HCC cells was markedly inhibited by 4MOD treatment (Figures 1(e) and 1(f)). Taken together, 4MOD can significantly inhibit the proliferation of liver cancer *in vitro.*

### 3.2. 4MOD Inhibits the Migration of HCC Cells

To ascertain the effect of 4MOD on HCC cells' migration, wound healing, and transwell migration assays were performed. After 24 or 48 h of creating the scratch wound, 4MOD treatment significantly inhibited wound healing (Figures 2(a) and 2(b)). Transwell migration experiments showed that the number of cells at the bottom of the upper chamber in 4MOD-treated groups was less than that in the 0 *μ*M group after 24 h of seeding (Figures 2(c) and 2(d)). Wound healing and transwell migration experiments revealed that 4MOD could significantly inhibit the migration of liver cancer.

### 3.3. 4MOD Induces Apoptosis of HCC Cells

To observe whether apoptosis was related to the anticancer effects of 4MOD in HCC, we detected the apoptotic ratio using flow cytometry. We found that 4MOD could induce apoptosis in liver cancer cells. The apoptosis rate of SK-HEP-1 cells without 4MOD treatment (0 *μ*M group) was 6.14%, while the apoptosis rate of SK-HEP-1 cells with 4MOD treatment (40 *μ*M group) was up to 50.9%. However, low concentration of 4MOD (20 *μ*M) had no impact on SK-HEP-1 cells apoptosis (Figure 3(a)). Similarly, the apoptosis rate of the 4MOD (20 *μ*M) group (40.6%) was significantly higher than that of the control (0 *μ*M) group (6.08%) and low concentration (10 *μ*M) group (6.74%) in HuH-7 cells (Figure 3(b)).

### 3.4. Differential Gene Expression Analysis

To understand the potential anticancer mechanisms of 4MOD in SK-HEP-1 cells, we performed RNA-Seq on control cells and treated cells using the Illumina Novaseq6000 system. Upon analysis, a total of 600 DEGs (387 up- and 213 downregulated genes) were identified between 4MOD-treated (20 *μ*M) groups and the control groups (0 *μ*M) (Figures 4(a) and 4(b)). Based on the absolute log2 fold change, the top 20 up and downregulated DEGs are shown in the heatmap (Figures 4(c) and 4(d)).

### 3.5. GO, KEGG, and GSEA Enrichment Analyses of DEGs

To further uncover the molecular mechanisms of 4MOD against HCC, GO, KEGG, and GSEA, enrichment analyses were performed on all DEGs. GO biological processes (BP) annotations showed that the DEGs mainly participated in the regulation of multicellular organismal processes, positive regulation of multicellular organismal processes, and muscle structure development (Figure 5(a)). GO cellular component (CC) annotations showed that the DEGs mainly focused on the extracellular matrix, the extracellular region part, and the transcription factor AP-1 complex (Figure 5(b)). GO molecular function (MF) annotations showed that the DEGs were associated with transcription factor binding, DNA-binding transcription factor activity, RNA polymerase II-specific and signaling receptor binding (Figure 5(c)). According to KEGG pathway enrichment analysis, DEGs were mainly enriched in the MAPK signaling pathway, IL-17 signaling pathway, and cytokine-cytokine receptor interaction (Figure 5(d)). The GSEA analysis showed that a number of DEGs were significantly related to MAPK signaling pathway (Figure 5(e)).

### 3.6. Transcriptome Validation by qRT-PCR

Considering that the MAPK pathway was the most significantly enriched pathway in this study, DEGs that participated in the regulation of the MAPK pathway were identified. The heatmap showed all of the DEGs involved in the regulation of the MAPK pathway, with GADD45G being the most significantly upregulated gene (Figure 6(a)). Ten of DEGs associated with MAPK pathway were further validated by qRT-PCR (Figure 6(b)). In HuH-7 cells, qRT-PCR results also revealed that 4MOD upregulated GADD45G mRNA expression (Figure 6(c)).

### 3.7. Downregulation of GADD45G Rescues the Regulation of Proliferation, Migration, and Apoptosis by 4MOD in HCC Cells

To explore whether 4MOD elicited anti-HCC activities by upregulating GADD45G expression *in vitro*, we transfected specific shRNA sequences into HCC cells to knockdown GADD45G expression. Our qRT-PCR data showed that shGADD45G transfection significantly reduced GADD45G expression (Figure 7(a)). We first examined whether downregulation of GADD45G could eliminate the inhibitory effects of 4MOD on HCC cell proliferation. Our CCK8 data revealed that GADD45G downregulation promoted cell viability in SK-HEP-1 and HuH-7 cells (Figures 7(b) and 7(c)). The migration ability of HCC cells transfected with shGADD45G plus 4MOD was examined by a wound healing assay. As expected, downregulation of GADD45G reversed 4MOD-mediated reduction of migration activity in HCC cells (Figures 7(d) and 7(e)). In addition, we further verified that 4MOD-induced apoptosis was partially inhibited by GADD45G downregulation (Figures 7(f) and 7(g)).

## 4. Discussion

HCC is a common malignant neoplasm with high morbidity and mortality rates. Although a variety of chemotherapeutic drugs are widely used, the high incidence of drug resistance has become the main reason for chemotherapy failure [18]. Consequently, it is necessary to explore more effective drugs with low toxicity against HCC.

Excessive proliferation, uncontrolled migration, and abnormal apoptosis are important malignant biological behaviors of tumor cells [19, 20]. It is well known that several natural herbal products exhibit remarkably anticancer effects by inhibiting tumor cells proliferation, migration, and inducing apoptosis. For decades, 4MOD has been known as a natural flavonoid compound with anti-inflammatory activity. Recently, 4MOD has been shown to inhibit tumor cells growth and migration, as well as to promote apoptosis [12, 13]. Mechanistically, 4MOD exerts anticancer effects on human bladder cancer through inactivating the AKT/ERK signaling pathway and inducing autophagy [12]. Nevertheless, the antitumor effects and mechanism of action of 4MOD against liver cancer remain unknown.

In this study, 4-Methoxydalbergione's anticancer effects and underlying mechanisms in HCC were explored. Our *in vitro* results showed that 4MOD repressed HCC cells proliferation and migration. Furthermore, flow cytometry analysis proved that high concentrations of 4MOD remarkably promoted tumor cell apoptosis. Therefore, our results demonstrated that 4MOD has anti-HCC activity and could be a valuable anticancer agent. However, it is necessary to validate these findings *in vivo*.

Studies have shown that many natural herbal products exert anticancer activity by interacting with multiple target genes and various signaling pathways [21, 22]. RNA-Seq analysis has become a mature tool for exploring the potential mechanisms of natural herbal products in cancer treatment and identifying candidate drug targets. In our study, RNA-Seq was performed to explore the anti-HCC molecular mechanism of 4MOD *in vitro*. In total, 600 target genes (387 up- and 213 down-regulated genes) were identified based on differential gene expression. Although these target genes need to be further validated, our study offers a valuable research direction for future functional studies. Moreover, we performed GO, KEGG, and GSEA analyses to uncover the anticancer mechanisms of 4MOD. According to the results of KEGG enrichment analysis, multiple molecular pathways were altered in SK-HEP-1 cells upon 4MOD treatment, including the MAPK signaling pathway.

The MAPK pathway is a common signaling pathway in human disease, including four main pathways: ERK, JNK, p38/MAPK, and ERK5 signaling [23, 24]. Abnormal activation of the MAPK signaling pathway can result in various cancers, including HCC [25]. Our RNA-Seq and qRT-PCR results showed a variety of abnormal expression genes related to the MAPK pathway, including GADD45G. These genes may influence the malignant biological behavior of HCC by regulating the activation of the MAPK pathway. GADD45G is a tumor suppressor gene, which is known to regulate cell proliferation through the MAPK pathway [16]. Evidence has shown that overexpression of GADD45G in tumor cells inhibits tumor proliferation and migration and promotes apoptosis [14–16, 26]. Our RNA-seq results revealed that 4MOD was able to upregulate GADD45G mRNA expression. We hypothesized that knockdown of GADD45G might promote the malignant biological behavior of HCC cells. We further verified that 4MOD could enhance GADD45G expression in HCC cell lines. After silencing the expression of GADD45G, the abilities of 4MOD to induce apoptosis and inhibit proliferation and migration were weakened in HCC cells. In short, 4MOD significantly inhibited the growth of human liver cancer cells *in vitro* by targeting GADD45G. However, our findings cannot explain the specific molecular mechanism underlying 4MOD-mediated GADD45G upregulation. Future studies will be needed to explore the specific molecular mechanisms involved.

## 5. Conclusions

Our results demonstrate for the first time that 4MOD could suppress proliferation and migration and promote apoptosis by targeting GADD45G in HCC cells. These results provide novel directions for exploring the drug therapy of liver cancer, implying that 4MOD may be used as a new antitumor agent in the future.

## Figures and Tables

**Figure 1:** 4MOD inhibits HCC proliferation. (a, b) Morphological changes of SK-HEP-1 and HuH-7 cells treated with different doses of 4MOD for 48 h (100x). (c, d) CCK-8 assay on SK-HEP-1 and HuH-7 cells treated with different doses of 4MOD at different times. (e, f) Colony formation assay on SK-HEP-1 and HuH-7 cells exposed to 0, 5 and 10 *μ*M of 4MOD for 48 h. The histogram shows statistical analysis for the colony numbers. ^*∗*^*p* <  0.05 and ^*∗∗∗*^*p* < 0.001, compared with control group (0 *μ*M).

**Figure 2:** 4MOD inhibits HCC migration. (a, b) Wound healing assay on SK-HEP-1 and HuH-7 cells treated with or without 4MOD for 24 and 48 h (40x). The histogram shows statistical analysis for the scratch area. (c, d) Transwell migration assay on SK-HEP-1 cells and HuH-7 cells treated with or without 4MOD for 48 h (100x). The histogram shows statistical analysis for the migration cells. ns, *p* ≥ 0.05, ^*∗*^*p* < 0.05, ^*∗∗*^*p* < 0.01, and ^*∗∗∗*^*p* < 0.001, compared with control group (0 *μ*M).

**Figure 3:** 4MOD induces apoptosis of HCC cells. (a) Flow cytometry on apoptosis rates of SK-HEP-1 cells exposed to 0, 20, and 40 *μ*M of 4MOD for 48 h. The histogram shows statistical analysis for the apoptotic cells. (b) Flow cytometry on apoptosis rates of HuH-7 cells exposed to 0, 10, and 20 *μ*M of 4MOD for 48 h. The histogram shows statistical analysis for the apoptotic cells. ns, *p* ≥ 0.05, ^*∗∗∗*^*p* < 0.001, compared with 0 *μ*M group.

**Figure 4:** Differential gene expression analysis between the 4MOD-treatment groups (20 *μ*M) and control groups (0 *μ*M) in SK-HEP-1 cells. (a) Volcano plot of DEGs. (b) Histogram of DEGs. (c) Heatmap of top 20 upregulated DEGs. (d) Heatmap of top 20 downregulated DEGs.

**Figure 5:** GO, KEGG and GSEA enrichment analyses of DEGs. (a) GO-BP annotations. (b) GO-CC annotations. (c) GO-MF annotations. (d) KEGG pathway enrichment analysis. (e) GSEA enrichment analysis.

**Figure 6:** Transcriptome validation by qRT-PCR. (a) Heatmap of DEGs involved in the regulation of MAPK pathway. GADD45G, the most significantly upregulated gene, was marked in the red box. (b) qRT-PCR validation on ten dysregulated genes involved in MAPK signaling pathway in SK-HEP-1 cells. (c) Expression levels of GADD45G were detected in 4MOD-treatment groups (10 *μ*M) and control groups (0 *μ*M) by qRT-PCR in HuH-7 cells. ^*∗*^*p* < 0.05, ^*∗∗*^*p* < 0.01, and ^*∗∗∗*^*p* < 0.001, compared with 0 *μ*M group.

**Figure 7:** 4MOD exerts anticancer effects by upregulating GADD45G expression in HCC. (a) The relative GADD45G mRNA expression was detected by qRT-PCR in shGADD45G-transfected cells. (b, c) SK-HEP-1 and HuH-7 cells were transfected with negative control (shNC) or shGADD45G, respectively. CCK8 was used to detect cell viability after treatment with or without 4MOD (20 *μ*M) for 48 h. (d) SK-HEP-1 was transfected with shNC or shGADD45G, respectively. Wound healing assay was used to detect cell migration after treatment with or without 4MOD (20 *μ*M) for 48 h. (e) HuH-7 was transfected with shNC or shGADD45G, respectively. Wound healing assay was used to detect cell migration after treatment with or without 4MOD (10 *μ*M) for 48 h. (f) SK-HEP-1 were transfected with shNC or shGADD45G, respectively. Flow cytometry was used to detect cell apoptosis after treatment with or without 4MOD (40 *μ*M) for 48 h. (g) HuH-7 was transfected with shNC or shGADD45G, respectively. Flow cytometry was used to detect cell apoptosis after treatment with or without 4MOD (20 *μ*M) for 48 h. ^*∗∗*^*p* < 0.01, ^*∗∗∗*^*p* < 0.001.

**Table 1:** Primer sequences used for qRT-PCR.

Genes	Primer sequence (5′-3′)
GADD45G	Forword: ACACAGTTCCGGAAAGCACA
	Reverse: TTTGGCTGACTCGTAGACGC

PDGFRA	Forword: TTGAAGGCAGGCACATTTACA
	Reverse: GCGACAAGGTATAATGGCAGAAT

JUND	Forword: TCATCATCCAGTCCAACGGG
	Reverse: TTCTGCTTGTGTAAATCCTCCAG

FOS	Forword: CACTCCAAGCGGAGACAGAC
	Reverse: AGGTCATCAGGGATCTTGCAG

HSPA1A	Forword: AACTCCACCATCCCCACC
	Reverse: CTCGCCCTCGTACACCTG

HSPA1B	Forword: TTTGAGGGCATCGACTTCTACA
	Reverse: CCAGGACCAGGTCGTGAATC

HSPA6	Forword: GATGTGTCGGTTCTCTCCATTG
	Reverse: CTTCCATGAAGTGGTTCACGA

NGFR	Forword: TGGCCTACATAGCCTTCAAGA
	Reverse: GAGATGCCACTGTCGCTGT

PGF	Forword: GAACGGCTCGTCAGAGGTG
	Reverse: ACAGTGCAGATTCTCATCGCC

RAC3	Forword: ATGTCCGTGCAAAGTGGTATC
	Reverse: CTCGGATCGCTTCGTCAAACA

GAPDH	Forword: CAGGAGGCATTGCTGATGAT
	Reverse: GAAGGCTGGGGCTCATTT

**Table 2:** Inhibitory concentration 50% (IC_50_) of 4MOD in HCC cells.

	SK-HEP-1 (*μ*M)	HuH-7 (*μ*M)
IC_50_-24 h	42.09 ± 1.77	31.16 ± 1.65
IC_50_-48 h	29.33 ± 0.33	22.83 ± 1.1
IC_50_-72 h	13.38 ± 0.37	13.95 ± 1.17

## Data Availability

The experiment data used to support the findings of this study are available from the corresponding author upon request.

## References

[1] Sung H., Ferlay J., Siegel R. L. (2021). Global cancer statistics 2020: GLOBOCAN estimates of incidence and mortality worldwide for 36 cancers in 185 countries. *CA: A Cancer Journal for Clinicians*.

[2] Wang H., Lu Z., Zhao X. (2019). Tumorigenesis, diagnosis, and therapeutic potential of exosomes in liver cancer. *Journal of Hematology & Oncology*.

[3] Tang W., Chen Z., Zhang W. (2020). The mechanisms of sorafenib resistance in hepatocellular carcinoma: theoretical basis and therapeutic aspects. *Signal Transduction and Targeted Therapy*.

[4] Luo H., Vong C. T., Chen H. (2019). Naturally occurring anti-cancer compounds: shining from Chinese herbal medicine. *Chinese Medicine*.

[5] Hassanalilou T., Ghavamzadeh S., Khalili L. (2019). Curcumin and gastric cancer: a review on mechanisms of action. *Journal of Gastrointestinal Cancer*.

[6] Kumar S., Chang Y. C., Lai K. H. (2021). Resveratrol, a molecule with anti-inflammatory and anti-cancer activities: natural product to chemical synthesis. *Current Medicinal Chemistry*.

[7] Guan F., Ding Y., Zhang Y., Zhou Y., Li M., Wang C. (2016). Curcumin suppresses proliferation and migration of MDA-MB-231 breast cancer cells through autophagy-dependent akt degradation. *PLoS One*.

[8] Maleki S. J., Crespo J. F., Cabanillas B. (2019). Anti-inflammatory effects of flavonoids. *Food Chemistry*.

[9] Kopustinskiene D. M., Jakstas V., Savickas A., Bernatoniene J. (2020). Flavonoids as anticancer agents. *Nutrients*.

[10] Pietta P. G. (2000). Flavonoids as antioxidants. *Journal of Natural Products*.

[11] Chan S. C., Chang Y. S., Wang J. P., Chen S. C., Kuo S. C. (1998). Three new flavonoids and antiallergic, anti-inflammatory constituents from the heartwood of Dalbergia odorifera. *Planta Medical*.

[12] Du H., Tao T., Xu S. (2021). 4-Methoxydalbergione inhibits bladder cancer cell growth via inducing autophagy and inhibiting akt/ERK signaling pathway. *Frontiers in Molecular Biosciences*.

[13] Li R., Xu C. Q., Shen J. X. (2021). 4-Methoxydalbergione is a potent inhibitor of human astroglioma U87 cells in vitro and in vivo. *Acta Pharmacologica Sinica*.

[14] Li T., Xu L., Teng J. (2020). GADD45G interacts with E-cadherin to suppress the migration and invasion of esophageal squamous cell carcinoma. *Digestive Diseases and Sciences*.

[15] Zhang X., Li Y., Ji J. (2021). Gadd45g initiates embryonic stem cell differentiation and inhibits breast cell carcinogenesis. *Cell Death & Disease*.

[16] Guo D., Zhao Y., Wang N. (2021). GADD45g acts as a novel tumor suppressor, and its activation suggests new combination regimens for the treatment of AML. *Blood*.

[17] Xu G., Zhang L., Ma A. (2015). SIP1 is a downstream effector of GADD45G in senescence induction and growth inhibition of liver tumor cells. *Oncotarget*.

[18] Huang A., Yang X. R., Chung W. Y., Dennison A. R., Zhou J. (2020). Targeted therapy for hepatocellular carcinoma. *Signal Transduction and Targeted Therapy*.

[19] Zou Y., Ye F., Kong Y. (2022). The single-cell landscape of intratumoral heterogeneity and the immunosuppressive microenvironment in liver and brain metastases of breast cancer. *Advanced Science*.

[20] Liu P., Wang Z., Ou X. (2022). The FUS/circEZH2/KLF5/feedback loop contributes to CXCR4-induced liver metastasis of breast cancer by enhancing epithelial-mesenchymal transition. *Molecular Cancer*.

[21] Pan J., Chen H., Guo B., Liu C. (2017). Understanding the molecular mechanisms underlying the effects of light intensity on flavonoid production by RNA-seq analysis in Epimedium pseudowushanense B.L.Guo. *PLoS One*.

[22] Yang Z., Zhang Q., Yu L., Zhu J., Cao Y., Gao X. (2021). The signaling pathways and targets of traditional Chinese medicine and natural medicine in triple-negative breast cancer. *Journal of Ethnopharmacology*.

[23] Plotnikov A., Zehorai E., Procaccia S., Seger R. (2011). The MAPK cascades: signaling components, nuclear roles and mechanisms of nuclear translocation. *Biochimica et Biophysica Acta (BBA) - Molecular Cell Research*.

[24] Pimienta G., Pascual J. (2007). Canonical and alternative MAPK signaling. *Cell Cycle*.

[25] Moon H., Ro S. W. (2021). MAPK/ERK signaling pathway in hepatocellular carcinoma. *Cancers*.

[26] Zhang L., Yang Z., Ma A. (2014). Growth arrest and DNA damage 45G down-regulation contributes to Janus kinase/signal transducer and activator of transcription 3 activation and cellular senescence evasion in hepatocellular carcinoma. *Hepatology*.

